# Efficacy of Postoperative Analgesia by Erector Spinal Plane Block after Lumbar Surgery: A Systematic Review and Meta-analysis of Randomized Controlled Trials

**DOI:** 10.1155/2022/3264142

**Published:** 2022-08-11

**Authors:** Xiao Xiao, Tingting Zhu, Lin Wang, Hongmei Zhou, Yanli Zhang

**Affiliations:** ^1^Department of Anesthesiology, The Second Hospital of Jiaxing, China; ^2^Department of Anesthesia Operating Room, The Second Hospital of Jiaxing, China

## Abstract

**Background:**

In recent years, erector spinae plane block (ESPB) has been increasingly used as a new regional block technique for postoperative analgesia; however, little is known on its benefits. Therefore, we performed a systematic review and meta-analysis to investigate the efficacy and safety of ESPB in lumbar spine surgery.

**Methods:**

Databases including PubMed, Embase, Cochrane Library, and Web of Science were systematically searched for randomized controlled trials (RCTs) comparing ESPB with no block in lumbar spine surgery until September 30, 2021. The primary outcome was opioid consumption after surgery. The Cochrane Collaboration's tool for assessing the risk of bias was used to evaluate the quality of included studies.

**Results:**

Fifteen RCTs involving 980 patients were included in the study. Opioid consumption 24 hours after surgery was significantly lower in the ESPB group standardized mean difference (SMD = −2.27, 95% confidence interval (95% CI) (-3.21, -1.32); *p* < 0.01). ESPB reduced pain scores at rest and on movement within 48 hours after surgery and the incidence of the postoperative rescue analgesia (RR = 0.32, 95% CI (0.31, 0.80); *p* = 0.02), while it significantly prolonged time to first rescue analgesia (SMD = 4.87, 95% CI (2.84, 6.90); *p* < 0.01). Moreover, significantly better patient satisfaction was associated with ESPB (SMD = 1.89, 95% CI (1.03, 2.74); *p* < 0.01).

**Conclusion:**

EPSB provides effective and safe postoperative analgesia after lumbar spine surgery.

## 1. Introduction

Severe postoperative pain after spinal surgery is a major factor affecting postoperative recovery and is associated with increased postoperative opioid use and prolonged hospitalizations [1]. The erector spinae plane block (ESPB) is a novel regional analgesia technique whereby local anesthesia (LA) is injected into the fascial plane deep into the erector spinae muscles and is considered a relatively safe and simple technique [2, 3]. First described in 2016 by Forero et al. [2], ESPB has been demonstrated to provide effective postoperative analgesia in thoracic and breast surgery [4]. A growing number of studies validated the benefits of ESPB, including reduced postoperative pain scores, postoperative opioid consumption, and postoperative nausea and vomiting (PONV) risk [4, 5]. In recent years, some randomized controlled trials (RCTs) [6–8] have been published on the use of ESPB after lumbar spine surgery; however, the robustness of the findings was questionable due to the limited sample size. Herein, we conducted a meta-analysis to explore the efficacy and safety of ESPB in adult patients who received general anesthesia (GA) for lumbar spine surgery. Our primary outcome was postoperative opioid consumption. Secondary outcomes included postoperative pain score, time to first rescue analgesia, number of patients requiring rescue analgesia, patient satisfaction, the length of hospitalization, and adverse reactions.

## 2. Methods

This systematic review and meta-analysis was based on the guidelines recommended by the Preferred Reporting Items for Systematic Reviews and Meta-Analyses (PRISMA) [9] and registered at the PROSPERO database (CRD42021276713).

### 2.1. Search Strategy

PubMed, Embase, the Cochrane Library, and Web of Science were systematically searched for relevant studies up to September 1, 2021, using the terms: (“Erector Spinae Plane Block” OR “Erector Spinae Plane Blocks” OR “Regional Anesthesia” OR “Regional Analgesia”) AND (“Lumbar Disc Disease” OR “Lumbar Spinal Surgery” OR “Lumbar surgery” OR “Lumbar fusion surgery” OR “Lumbar discectomy”). No restriction was made with respect to language. Additionally, reference lists of studies meeting the above criteria were reviewed to identify additional relevant articles that could be included.

### 2.2. Study Selection Criteria

Three authors (Z. YL., XX., and W. L.) independently searched the literature, and any point of disagreement was solved by a discussion with a fourth author (Z.TT). Search results were imported into EndNote X9, and duplicates were removed. All published RCTs with full text available that compared ESPB with no block after lumbar spine surgery were included in this study. Trials that did not report postoperative opioid consumption were excluded. Letters, retrospective studies, case reports, reviews, incomplete clinical trials, studies without control groups, studies without full text, and conference abstracts were also excluded.

### 2.3. Data Extraction and Quality Assessment

Two authors (Z. YL. and X.X.) extracted the following information: first author, published year, type of surgery, techniques, concentration and volume of local anesthesia, postoperative analgesia, rescue analgesia, postoperative pain scores, postoperative opioid analgesic consumption, adverse reactions, etc.

To facilitate data analysis, we calculated the median and interquartile range (IQR) as described by Luo et al. [10] and the standard deviation (SD) as defined by Wan et al. [11]. For studies where the original data were presented in graphical format, the GetData graph digitizer was used to extract numerical data. The pain scores 48 hours after surgery at rest and on movement were extracted. If not otherwise stated, we assumed that pain scores were assessed at rest. Methodological quality assessment was independently done by the two authors (Z. YL. and X.X.) using Cochrane Collaboration's tool for assessing risk of bias. We evaluated the quality of all studies based on seven aspects: trials were considered low quality if at least one category was graded “high risk of bias” while trials were considered high quality if the randomization and allocation concealment were both graded “low risk of bias,” and other items were graded “low risk of bias” or “uncertain risk of bias.” Finally, trials were considered moderate quality if no criteria for high or low risk of bias were met.

### 2.4. Statistical Analysis

Review Manager (RevMan, version 5.3, The Nordic Cochrane Centre, The Cochrane Collaboration, Copenhagen, Denmark) was used for this meta-analysis. For continuous data, the standardized mean difference (SMD) and 95% confidence intervals (CI) were calculated using random-effect model while for dichotomous data, the Mantel-Haenszel method was used to calculate the relative ratio (RR) and 95% CIs. The *I*^2^ statistic was used to quantify statistical heterogeneity. If significant heterogeneity was observed (*I*^2^ < 50%), a fixed-effect model was adopted; otherwise, a random-effect model was applied. *p* < 0.05 (2-sided) was considered statistically significant. Funnel plots were used to evaluate the publication bias.

## 3. Results

### 3.1. Results of Literature Search and Characteristics

The initial search yielded 718 references, with no additional records from other sources. The records were imported into EndNote X9, and 524 unqualified records were excluded. After reading the title and abstracts, only 21 articles remained. Finally, 15 trials involving 980 participants met the inclusion criteria. A flowchart of the literature screening process is shown in Figure 1. The Cochrane Collaboration risk of bias tool (Figure 2) was used to determine the risk of bias in included studies.

Of the 15 trials included [6–8, 12–23], one [17] involved free-hand ESPB, while the others [6–8, 12–16, 18–23] were ultrasound-guided (USG-guided) ESPB. The main local anesthetics used included bupivacaine [6–8, 12–14, 16, 18, 19], ropivacaine [20–23], levobupivacaine [15], and mixtures of bupivacaine and lidocaine [17]. The features of the included trials are shown in Table 1.

### 3.2. Primary Outcomes

All trials [6–8, 12–23] reported postoperative opioid consumption; however, only one trial [13] reported opioid consumption 8 hours after surgery. The pooled analysis showed that ESPB could reduce 4 to12 hours (SMD = −2.46, 95% CI (−3.62, −1.29); *p* < 0.01; Figure 3), 24 hours (SMD = −2.27, 95% CI (−3.21, −1.32); *p* < 0.01; Figure 4), and 48 hours (SMD = −0.83, 95% CI (−1.05, −0.60); *p* < 0.01; Figure 5) postoperative opioid consumption.

### 3.3. Secondary Outcomes

Moreover, ESPB significantly reduced postoperative pain scores at rest (PACU: SMD = −1.86, 95% CI (-2.59, -1.13); *p* < 0.01; 2 h: SMD = −1.73: 95% CI (-2.70, -0.75); *p* < 0.01; 4 h: SMD = −1.38, 95% CI (-2.15, 0.61); *p* < 0.01; 6 h: SMD = −2.26, 95% CI (-3.54, -0.99); *p* < 0.01; 12 h: SMD = −0.69, 95% CI (-1.14, -0.24); *p* < 0.01; 24 h: SMD = −0.52, 95% CI (-0.75, -0.29); *p* < 0.01; 48 h: SMD = −0.33, 95% CI (-0.61, -0.06); *p* = 0.02) and on movement (PACU: SMD = −1.31, 95% CI (-2.14, -0.48); *p* < 0.01; 4 h: SMD = −1.20, 95% CI (-2.31, -0.09); *p* = 0.03; 6 h: SMD = −8.24, 95% CI (-13.40, -3.08); *p* < 0.01; 12 h: SMD = −3.21, 95% CI (-5.67, -0.75); *p* = 0.02; 24 h: SMD = −1.05, 95% CI (-1.94, -0.17); *p* = 0.02; 48 h: SMD = −0.70, 95% CI (-1.05, -0.35); *p* < 0.01). Importantly, ESPB could significantly prolong time to first rescue analgesia (SMD = 4.87, 95% CI (2.84, 6.90); *p* < 0.01), reduce intraoperative opioid consumption (SMD = −1.48, 95% CI (-2.35, -0.6); *p* < 0.01), and reduce the number of patients requiring rescue analgesia (RR = 0.32, 95% CI (0.13, 0.80); *p* = 0.02). Furthermore, ESPB could reduce the incidence of PONV (RR = 0.35, 95% CI (0.22, 0.55); *p* < 0.01), shorten the length of hospitalization (MD = −1.80, 95% CI (-3.21, -0.39); *p* = 0.01), and improve patient satisfaction (SMD = 1.89, 95% CI (1.03, 2.74); *p* < 0.01). Detailed information on the secondary outcomes is presented in Table 2.

### 3.4. Quality Assessment and Publication Bias

All trials described the random sequence generation methodology, and six trials [7, 8, 10, 13, 20–22] described allocation concealment methods used. Four trials [15, 17–19] described the blinding of participants and personnel, while one trial [13] did not mention blinding of outcome assessment. Complete data were available in all included studies, with no selective reporting or bias. Quality assessment results are displayed in Figure 2. No publication bias was found by visual inspection of funnel plots (Figure 6).

## 4. Discussion

Herein, we sought to investigate whether ESPB offered superior analgesia after lumbar spine surgery by pooling data of 15 RCTs that involved 980 participants. Importantly, we found that ESPB could significantly reduce postoperative opioid consumption in this patient population. Additionally, ESPB helped prolong the time to first rescue analgesia and reduced postoperative acute pain scores, intraoperative opioid consumption, the number of patients requiring postoperative rescue analgesia, the incidence of PONV, and shortened the length of hospitalization. These parameters contributed to better patient satisfaction. Given that the pooled estimates showed a high degree of heterogeneity, the quality of evidence of our outcomes was low to moderate.

The ESPB technique involves the injection of LA into the fascial planes between the erector spinae muscles and the transverse process. The mechanisms underlying the efficacy of ESPB remain unclear. Few studies have examined LA diffusion in ESPB and have not suggested an acceptable predictable diffusion [24]. Potential mechanisms of ESPB have been proposed: during ultrasound-guided ESPB, the local anesthetic drug has been found to spread from the injection site to the three upper vertebral body planes and four lower caudal paravertebral planes [25]. Interestingly, unilateral ESPB has been shown to exert a contralateral blockade effect, which may be accounted for by the spread of local anesthetic drug in the epidural membrane [26–28]. In addition, some evidence suggested that LA had dorsal branch diffusion [29]. Furthermore, it has been reported that ESPB can be used in posterior spinal surgery, possibly exerting analgesic effects by blockade of the posterior ramus of the spinal nerve [15]. Moreover, in recent years, ESPB has been evolving as an effective technique that can significantly reduce the risk of spinal cord or nerve roots injury and has huge prospects in replacing epidural analgesia for postoperative analgesia.

Severe postoperative pain associated with lumbar spine surgery is an important factor affecting the recovery of patients. Current evidence demonstrated that implementing Enhanced Recovery After Surgery (ERAS) programs after lumbar spine surgery may improve functional recovery and reduce the length of hospitalization, opioid consumption, complications, and unplanned readmission rate [30]. Postoperative analgesia is an important part of ERAS programs. In recent years, the implementation of ESPB has been documented to exert an effective postoperative analgesic effect, especially with ultrasound guidance [31–34]. Two recent meta-analyses [35, 36] have demonstrated the efficacy of ESPB for postoperative analgesia; however, they included fewer randomized controlled trials, smaller sample sizes, and significant heterogeneity in their results.

Herein, we demonstrated that ESPB reduced postoperative opioid consumption, which objectively reflected the efficacy of ESPB in postoperative analgesia. In this regard, ESPB could significantly lower pain scores during the first postoperative 48 hours at rest and on movement, but not the postoperative 2-hour pain score on movement. This finding may be accounted for by a high dose of rescue analgesia administered within 2 hours after surgery which lowered the pain scores. Moreover, few trials have evaluated postoperative 2-hour pain scores on movement. The traditional methods of postoperative analgesia rely mainly on postoperative opioid-based patient-controlled intravenous analgesia (PCIA). However, patients may experience adverse reactions, such as nausea and vomiting, dizziness, and constipation, while some patients even give up opioid-based PCIA. Side effects caused by postoperative opioid consumption lead to poor postoperative experience and low patient satisfaction and are not conducive to rapid recovery [37]. Alleviating acute postoperative pain is an important part of ERAS. In this regard, we found that ESPB could significantly reduce the length of hospitalization, which meets the requirements of ERAS. In addition, reducing the incidence of PONV in this patient population may improve satisfaction rates.

In recent years, ultrasound-guided ESPB has been increasingly used during clinical practice, and most of the trials (*n* = 14/15) included in our study used ultrasound-guided ESPB. In one study where intraoperative freehand bilateral ESPB was used [17], the authors documented significant benefits in terms of postoperative opioid consumption, time to first rescue analgesia, the number of rescue analgesia, and postoperative length of hospital stay. Importantly, freehand ESPB was simpler and safer, reduced serious complications, and did not require additional time to preparation compared with ultrasound-guided might provide a new idea for analgesia after lumbar surgery.

In one [19] of the included studies, the effects of ESPB in reducing the incidence of chronic pain after surgery were investigated. However, fewer cases with postoperative chronic pain were present in the ESPB group which could explain for the absence of statistically significant difference. However, in a pooled analysis of case reports by Viderman and Sarria-Santamera [38], effective pain relief was reported in 43 patients with documented chronic severe pain that underwent ESPB, suggesting that ESPB may be a new approach for the treatment of chronic pain.

The literature contains limited information on complications associated with ESPB. Tulgar et al. [39] reported bilateral postoperative quadriceps weakness in a 29-year-old patient that underwent bilateral ESPB for cesarean section and myomectomy. To the best of our knowledge, no block-related complications such as spinal nerve injury, lower extremity sensory or motor dysfunction, local anesthetic toxicity, and infection have been documented. Nonetheless, high-quality multicenter studies with large sample sizes are required to confirm the safety of ESPB.

This study has the following limitations. First, significant heterogeneity in the ESPB procedure was observed as different local anesthetics and methods were used in the included studies to evaluate acute pain. Furthermore, opioid consumption and pain scores were not presented as means and standard deviation but as medians and interquartile range or graphs. In addition, different types of opioids for analgesia accounted for high interstudy heterogeneity, and most of the outcomes had high heterogeneity. Moreover, a relatively small number of studies were included, and their quality was not high. In certain severe clinical situations [40–46], the effectiveness and safety of ESPB still need to be evaluated.

In conclusion, ESPB is effective and safe for postoperative analgesia after lumbar spine surgery. ESPB can reduce postoperative opioid consumption, improve patient satisfaction, and shorten the length of hospitalization. However, more high-quality trials are needed to substantiate our findings.

## Figures and Tables

**Figure 1:** PRISMA flow diagram of the literature selection. Records excluded during screening step: no postoperative opioid consumption, letters, retrospective studies, case reports, reviews, incomplete clinical trials, studies without control groups, studies without full text, and conference abstracts were also excluded.

**Figure 2:** Methodological quality and bias risk in included trials. Green, yellow, and red represent low, unclear, and high risk of bias, respectively.

**Figure 3:** Forest plots of opioid consumption 4 to12 hours after surgery.

**Figure 4:** Forest plots of opioid consumption 24 hours after surgery.

**Figure 5:** Forest plots of opioid consumption 48 hours after surgery.

**Figure 6:** Funnel plots detecting publication bias.

**Table 1:** The features of the included trials.

Author/year	Participants (*n*)	Age	Type of surgery	Techniques	ESPB group	Control group	Postoperative analgesia	Rescue analgesia
Ciftci et al. (2021) [6]	60	18–65 years	1-level lumbar discectomy and hemilaminectomy surgery	USG-guided ESPB	40 mL of 0.25% bupivacaine	No block	PCIA fentanyl, 1 g paracetamol every 6 hours	Meperidine (0.5 mg/kg)
Eskin et al. (2020) [7]	80	18–80 years	1- or 2-level lumbar decompression surgery	USG-guided ESPB	20 mL of 0.25% bupivacaine	No block	PCIA tramadol	Meperidine (0.5 mg/kg)
Elgebaly et al. (2019) [8]	60	18–60 years	2-level lumbar spondylolisthesis (L3-L5)	USG-guided ESPB	20 mL of 0.25% bupivacaine	Sham blocks (20 ml normal saline)	Paracetamol 1 gm/6 hours and ketorolac 30 mg loading dose then 15 mg/8 hours	Morphine 0.1 mg/kg iv. VAS > 30
Goel et al. (2021) [12]	100	18–78 years	1-level transforaminal lumbar interbody fusion surgery	USG-guided ESPB	20 mL of 0.25% bupivacaine	No block	1 gm paracetamol iv. Sixth hourly, 30 mg iv. ketorolac eighth hourly, pregabalin capsule 75 mg once a day	Fentanyl 1 mcg/kg iv. VAS ≥ 5
Siam et al. (2020) [13]	30	>18 years	Lumbar spine surgery	USG-guided ESPB	20 mL of 0.25% bupivacaine	Ketorolac 0.75 mg/kg and paracetamol 10 mg/kg	—	0.5 mg/kg peridine VAS > 4
Singh et al. (2019) [14]	40	18–65 years	Lumbar spine surgery	USG-guided ESPB	20 mL of 0.5% bupivacaine	No block	iv. diclofenac 1.5 mg/kg every 8 hours	iv. morphine 3 mg on demand or NRS≧4
Finnerty and Buggy (2021) [15]	140	18–65 years	2-level lumbar spine surgery	USG-guided ESPB	20 mL of 0.25% levobupivacaine	20 mL of normal saline 0.9%	iv. ketorolac 30 mg every 8 hourly, PCIA morphine	iv. Morphine VAS ≥ 4
Yayik et al. (2019) [16]	60	18–65 years	1- or 2-level open lumbar decompression surgery	USG-guided ESPB	20 mL of 0.025% bupivacaine	No block	400 mg IV ibuprofen 12 hourly; PCIA tramadol	25 mg pethidine VAS ≥ 4
Yeşiltaş et al. (2021) [17]	56	>18 years	Open posterior instrumentation and fusion	Free-hand ESPB	20 mL (1 : 1) mixture solution of 0.25% bupivacaine and 1.0% lidocaine	Sham blocks (20 mL physiological saline)	iv. 1 mg/kg tramadol, 1 g paracetamol	25 mg pethidine VAS ≥ 4
Yörükoğlu et al. (2021) [18]	54	18–65 years	1-level lumbar microdiscectomy	USG-guided ESPB	20 mL of 0.25% bupivacaine	Sham blocks (20 mL normal saline)	Tramadol (100 mg) and paracetamol (1 g), PCIA morphine	Tenoxicam 20 mg IV (NRS was >3)
Yu et al. (2021) [19]	80	26-67 years	1-level lumbar fracture	USG-guided ESPB	30 mL of 0.25% bupivacaine	Sham blocks (normal saline)	PCIA sufentanil and flurbiprofen	im. pethidine (NRS was >4)
Zhang et al. (2021) [20]	60	18–75 years	Lumbar spine surgery	USG-guided ESPB	25 mL of 0.3% ropivacaine	No block	PCIA morphine	PCIA bolus
Zhang et al. (2021) [21]	60	20–75 years	Open posterior lumbar spinal fusion surgery	USG-guided ESPB	20 mL 0.4% ropivacaine	Sham blocks	iv. flurbiprofen 300 mg, PCIA sufentanil	PCIA bolus
Zhang et al. (2020) [22]	60	18–80 years	Open posterior lumbar spinal fusion surgery	USG-guided ESPB	25 mL of 0.3% ropivacaine	No block	PCIA morphine	PCIA bolus
Zhu et al. (2021) [23]	40	45–70 years	Lumbar fusion	USG-guided ESPB	20 mL of 0.375% ropivacaine	Sham blocks (normal saline)	iv. sufentanil 5 *μ*g, flurbiprofen 50 mg, PCIA oxycodone	iv. sufentanil 5 *μ*g

**Table 2:** Secondary outcomes of RCTs included in meta-analysis.

Outcomes	Studies include	RR or SMD 95% CI	*p* value for statistical significance	*p* value for statistical heterogeneity	*I* ^2^ test for heterogeneity
VAS/NRS scores at the PACU (at rest)	9	-1.86 (-2.59, -1.13)	<0.01	<0.01	93%
VAS/NRS scores at the PACU (on movement)	3	-1.31 (-2.14, -0.48)	<0.01	<0.01	82%
VAS/NRS scores at 2 h (at rest)	7	-1.73 (-2.70, -0.75)	<0.01	<0.01	95%
VAS/NRS scores at 2 h (on movement)	2	-1.88 (-4.04, 0.27)	0.09	<0.01	95%
VAS/NRS scores at 4 h (at rest)	8	-1.38 (-2.15, 0.61)	<0.01	<0.01	94%
VAS/NRS scores at 4 h (on movement)	3	-1.20 (-2.31, -0.09)	0.03	<0.01	91%
VAS/NRS scores at 6 h (at rest)	8	-2.26 (-3.54, -0.99)	<0.01	<0.01	96%
VAS/NRS scores at 6 h (on movement)	3	-8.24 (-13.40, -3.08)	<0.01	<0.01	98%
VAS/NRS scores at 12 h (at rest)	9	-0.69 (-1.14, -0.24)	<0.01	<0.01	83%
VAS/NRS scores at 12 h (on movement)	5	-3.21 (-5.67, -0.75)	0.02	<0.01	94%
VAS/NRS scores at 24 h (at rest)	14	-0.52 (-0.75, -0.29)	<0.01	<0.01	66%
VAS/NRS scores at 24 h (on movement)	7	-1.05 (-1.94, -0.17)	0.02	<0.01	94%
VAS/NRS scores at 48 h (at rest)	7	-0.33 (-0.61, -0.06)	0.02	0.04	51%
VAS/NRS scores at 48 h (on movement)	5	-0.70 (-1.05, -0.35)	<0.01	0.07	53%
Time to first rescue analgesic	9	4.87 (2.84, 6.90)	<0.01	<0.01	98%
Intraoperative opioid consumption	8	-1.48 (-2.35, -0.6)	<0.01	<0.01	94%
Number of patients rescue analgesia (*n*)	10	0.32 (0.13, 0.80)	0.02	<0.01	97%
PONV (postoperative nausea and vomiting)	13	0.35 (0.22, 0.55)	<0.01	0.27	18%
The length of hospitalize	5	-1.80 (-3.21, -0.39)	0.01	<0.01	97%
Patient satisfaction	5	1.89 (1.03, 2.74)	<0.01	<0.01	92%

## Data Availability

The data used to support the findings of this study are available from the corresponding author upon request.
